# T cell immunohistochemistry refines lung transplant acute rejection diagnosis and grading

**DOI:** 10.1186/1746-1596-8-168

**Published:** 2013-10-14

**Authors:** Lin Cheng, Haizhou Guo, Xinwei Qiao, Quan Liu, Jun Nie, Jinsong Li, Jianjun Wang, Ke Jiang

**Affiliations:** 1 Department of Anesthesiology, Union hospital, Tongji Medical College, Huazhong University of Science and Technology, Wuhan, China; 2 Department of Thoracic Surgery, The First Affiliated Hospital, Zhengzhou University, Zhengzhou, China; 3 Department of Thoracic Surgery, Union hospital, Tongji Medical College, Huazhong University of Science and Technology, No.1277 Jiefang Avenue, Wuhan 430022, Hubei Province, P. R. China; 4 Department of Cardiovascular Surgery, Second Affiliated Hospital, Harbin Medical University, Harbin, China

**Keywords:** Lung transplantation, Immunohistochemistry, T lymphocyte

## Abstract

**Objective:**

Lung transplant volume has been increasing. However, inaccurate and uncertain diagnosis for lung transplant rejection hurdles long-term outcome due to, in part, interobserver variability in rejection grading. Therefore, a more reliable method to facilitate diagnosing and grading rejection is warranted.

**Method:**

Rat lung grafts were harvested on day 3, 7, 14 and 28 post transplant for histological and immunohistochemical assessment. No immunosuppressive treatment was administered. We explored the value of interstitial T lymphocytes quantification by immunohistochemistry and compared the role of T cell immunohistochemistry with H&E staining in diagnosing and grading lung transplant rejection.

**Results:**

Typical acute rejection from grade A1 to A4 was found. Rejection severity was heterogeneously distributed in one-third transplanted lungs (14/40): lesions in apex and center were more augmented than in the base and periphery of the grafts, respectively. Immunohistochemistry showed profound difference in T lymphocyte infiltration among grade A1 to A4 rejections. The coincidence rate of H&E and immunohistochemistry was 77.5%. The amount of interstitial T lymphocyte infiltration increased gradually with the upgrading of rejection. The statistical analysis demonstrated that the difference in the amount of interstitial T lymphocytes between grade A2 and A3 was not obvious. However, T lymphocytes in lung tissue of grade A4 were significantly more abundant than in other grades.

**Conclusions:**

Rejection severity was heterogeneously distributed within lung grafts. Immunohistochemistry improves the sensitivity and specificity of rejection diagnosis, and interstitial T lymphocyte quantitation has potential value in diagnosing and monitoring lung allograft rejection.

**Virtual slides:**

The virtual slides for this article can be found here: http://www.diagnosticpathology.diagnomx.eu/vs/1536075282108217.

## Introduction

To transplantation pathologists, there are still many difficulties and controversies in diagnosing and grading lung transplant rejection [1]. The transbronchial lung puncture biopsy is one of the accepted standards. Histological results are widely used in diagnosing and monitoring pulmonary graft rejection. In clinic, it is reasonable to modify the therapeutic strategy according to histological report. Generally, patients with positive histological results demonstrate good response to immunotherapy. Interestingly, patients with symptoms but negative biopsy results also benefit from immunotherapy such as intensive corticosteroid therapy. The reasons for this phenomenon are yet to be known. However, this phenomenon indicates that, to a certain extent, there may be potential ongoing rejection that is not discovered [2]. Therefore, a more reliable method to diagnose the rejection in transplanted lung is warranted.

Although the International Society for Heart and Lung Transplantation has published detailed classification of lung graft rejection, there are still many difficulties in clinical practice. This guideline emphasizes that at least five gassy lung tissue samples are needed for diagnosis. The diagnostic accuracy can be improved with increasing biopsy frequency which, however, may cause more complications associated with needle biopsy. Furthermore, perivascular mononuclear cell infiltration is not specific for acute rejection. The same changes also happen in other diseases, such as cytomegalovirus infection and post-transplantation lymphopoiesis, and thus lead to difficult rejection diagnosis. It is of great importance that pathologic diagnosis for the same lesion varies among different centers and even among pathologists in the same center [3-5]. Given all that, there are inaccuracy and uncertainty during the diagnostic process for lung transplant rejection.

A number of factors contribute to this situation. Insufficient graft tissue collection by needle biopsy, limited diagnostic information from routine H&E staining, pathologists’ different perceptions about the standard of rejection status and selective bias with diagnosis all affect diagnostic accuracy. Recently, Fabio Tavora and colleagues studied lung tissue sections by immunohistochemistry (IHC). They found that T lymphocyte infiltration was helpful to diagnosing and grading rejection [6]. Additionally, further information from other methods can also help improve diagnostic accuracy.

In this study, histological changes in the whole transplanted lungs, instead of graft tissues harvested by needle biopsy, were examined, which enabled us to understand the full extent of rejection. We also performed CD3, CD4 and CD8 IHC to detect the variation of T cells in lung grafts, and evaluated the value of quantitating interstitial T lymphocytes by IHC in rejection diagnosis and grading. We found that T cell IHC may provide additional information to avoid interobserver variability.

## Material and methods

### Animals

Specific pathogen free, male Brown Norway (BN) and Lewis (LEW) rats weighing 250-300 g were used. All animals were housed in the specific pathogen free facility (Tongji Medical College, Huazhong University of Science and Technology, Wuhan, China) and had access to water and food ad libitum. This study was approved by the Institutional Animal Research Committee of Union Hospital, Tongji Medical school, Huazhong University of Science and Technology. All animals received adequate care in accordance with the National Institutes of Health Guide for the Care and Use of Laboratory Animals.

### Orthotopic left lung transplantation

Left lung from LEW rats were orthotopicly implanted into LEW (syngeneic control, n = 40) or BN recipients (allogeneic, n = 40) as described before [7]. Lung grafts were harvested from CO_2_ euthanized recipients on day 3, 7, 14 and 28 after transplantation for histological and immunohistochemical analyses. Lungs from twelve-week-old male naïve LEW rats were used as naive control. All recipient animals received no immunosuppression.

### Histology and immunohistochemistry

Lung explants were was fixed with 10% formalin at room temperature for 8 h and embedded in paraffin. 4 μm sections or 5 μm sections were used for H&E staining or immunohistochemistry, respectively [8]. Primary anti-rat CD3, CD4 and CD8 (Bioss Inc) were used to detect T cells immunohistochemically, with appropriate irrelevant IgG as isotype control.

A microscope (BX51, Olympus) with camera (Axio Cam MRc, Carl Zeiss) and Image-Pro Plus 6.0 for windows (Media Cybernetics) analysis program were used for morphometric analysis. All measurements were performed on 3 random sections from each graft. All analyses were done by two independent and blinded reviewers, and the scores assigned were determined by consensus. The diagnoses of lung rejection were according to the grading standards of lung transplantation rejection formulated by the International Society for Heart and Lung Transplantation in 2006 [9].

### Statistical analysis

The concordance was quantified by the Kapper statistic, which ranges between -1.0 (perfect disagreement) and +1.0 (perfect agreement), with 0 representing chance agreement [10]. A weighted kapper (Kw) was computed for tables with more than 2 strata. A 2-tailed P values less than 0.05 were considered statistically significant. One-way repeated measures analysis of variance followed by t-test was used within the group. Statistical analysis was performed with SPSS version 13.0 software (Chicago, IL, USA).

## Results

### Histological heterogeneity in acutely rejected lung allografts

To explain the discrepancy between the biopsy and clinical outcomes, we proposed that histological heterogeneity might exist in lung allografts. To test this hypothesis, we first established LEW to BN lung transplantation model. As expected, acute rejection at A1-A4 occurred to all allotransplants (Figures 1 and 2). In general, the lung rejection was at grade 0-1 at day 3, grade 1-2 at day 7, grade 2-3 at day 14, and mainly above grade 3 during the second week after operation.

**Figure 1:** **The acute rejection of different levels in transplanted lung tissue. A**: grade A1 rejection; **B**: grade A2 rejection; **C**: grade A3 rejection; **D**: grade A4 rejection. **(A**-**C)** H&E, x200; **(D)** H&E, x400.

**Figure 2:** **Allografts at different time point post transplantation. A**: day 3; **B**: day 7; **C**: day 14; **D**: day 28. The left lung was transplanted and the right was native.

We found that 14 of 40 transplants showed heterogeneity of acute rejection within the allografts: the apex was more severely injured comparing with the base of lung transplants. Grossly, the focal pulmonary atelectasis generally occurred in the 14 lung apexes (Figure 3). In rejection of grade 3 and 4, the foci in apex merged with each other, accompanied by extensive blood extravasation that spread towards the base of lung allografts. Microscopy further confirmed that the intensities of rejection were different in different parts of lung allografts with rejection in the apex being more augmented than in the base and more in the center than in the periphery. Regarding rejection grading, difference of 1 and 2 between the apex and the base of lung allografts existed in 7 and 7 allografts (Table 1).

**Figure 3:** **The heterogeneous rejection 3 days post transplant.** The extravasated blood and foci of pulmonary atelectasis in the apex of left lung **(A)**. Histological and immnunohistochemical examination demonstrated grade A1 rejection in apex **(B**,**C)** and little evidence for acute rejection in the base of lung **(D)**. **C**-**D**: H&E, x200. **B**: CD3 IHC, x200.

**Table 1:** The heterogeneity of rejection in distribution within allografts

**Difference in grading**	**Grades**	**Number**	**Sum**
1 grade	A0-A1	2	7
	A1-A2	3	
	A2-A3	2	
2 grade	A0-A2	3	7
	A1-A3	3	
	A2-A4	1	

### T cell detection with CD4 and CD8 immunohistochemical staining may modify the classification of rejection

Grade A1 rejection, lymphocytes invading the alveolar septa in grades A2 and A3, and mononuclear cells in/under bronchial epithelium, are often overlooked with H&E staining. In contrast, T cell IHC possesses the advantage of clear background that makes it easier to diagnose and grade rejections. To evaluate the feasibility and justification of facilitating rejection evaluation with T cell IHC, tissue sections from different parts of the transplants were stained with CD4 and CD8 antibodies (Figure 4). CD4 and CD8 T cells in the grafts showed diffused distribution around the vessels or bronchi, which indicated ongoing rejection. IHC results helped revise grading of rejection in certain cases (Table 2). There was little difference in diagnosing and grading of graft rejection between H&E and IHC, with coincidence rate of the two methods being 77.5% and the overall weighted kw value being 0.688 (p < 0.001).

**Figure 4:** **CD4 and CD8 IHC in lung transplant rejection diagnosis and grading.** Tissue sections were immnunohistochemically stained with CD4 and CD8 antibodies and showed contrast against the background. **A**: grade A1 rejection; **B**: grade A2 rejection; **C**: grade A3 rejection; **D**: grade A4 rejection. (x200).

**Table 2:** Difference in diagnosing and grading rejection by H&E and IHC

**IHC**	**A0**	**A1**	**A2**	**A3**	**A4**
**HE**					
A0	35	4	3	0	0
A1	2	5	2	0	0
A2	1	2	6	2	0
A3	0	0	2	7	0
A4	0	0	0	0	9

Gray-shaded boxes highlight specimens graded the same during H&E and IHC.

IHC also revealed that T lymphocytes in acutely rejected lung transplants accumulated around the bronchovascular bundles and adjacent tissue. Furthermore, T lymphocytes in interstitial, that was lack of bronchovascular bundles, were also more in allografts comparing with normal lung tissue. The amount of T cells showed a positive correlation with the grading of rejection (Figure 5). Statistical analysis demonstrated that difference in interstitial T lymphocyte quantitation between grade A2 and A3 was not significant (P_CD3_ = 0.52, P_CD4_ = 0.93, P_CD8_ = 0.18). However, the T lymphocytes in grade A4 were significantly more than those in other grades (P_CD3_ = 0.08, P_CD4_ = 0.02, P_CD8_ = 0.03) (Figure 6).

**Figure 5:** **Interstitial cellular infiltration.** IHC showed interstitial CD3 T cell amount positively correlated with rejection severity with a better contrast than H&E staining. **A**: grade A0 rejection, **B**: grade A1 rejection, **C**: grade A2 rejection, **D**: grade A3 rejection. (x200).

**Figure 6:** **The differences of interstitial T lymphocytes in lung tissue between different rejection grades.** CD3 (P_A0-A1_ = 0.43, P_A1-A2_ = 0.02, P_A2-A3_ = 0.52, P_A3-A4_ = 0.03); CD4 (P_A0-A1_ = 0.06, P_A1-A2_ = 0.22, P_A2-A3_ = 0.93, P_A3-A4_ = 0.02); CD8 (P_A0-A1_ = 0.00, P_A1-A2_ = 0.02, P_A2-A3_ = 0.18, P_A3-A4_ = 0.03). Control: the normal lung tissue; A0-A4: the rejections in different intensity grades. Notes: The rejection grades were the final diagnoses based on the diagnostic standards of the International Society of Heart and Lung.

## Discussion

### Heterogeneity of lung allograft acute rejection

In this study, 14 of 40 acutely rejected allografts showed heterogeneous pathology within the transplants. Among them, the lesions in apex and center were more augmented than in the base and periphery of lungs, respectively.

Tsuyoshi et al. investigated 73 specimens by transbronchial biopsies and found rejection heterogeneity in 40 of 73 human lung recipients, among whom the upper lobes were higher graded in 35% (14/40) and the lower lobes were higher graded in 65% (26/40) [11]. Physiologically, the lower lobe receives greater blood flow than upper lobe [12]. This hemodynamic state may play some role in predisposing to the perivascular mononuclear infiltrating of acute rejection. Since rats are usually in prone position, blood supply is heterogeneously distributed in the lung, which probably results in heterogeneous acute rejection.

One-third cases in this study suffered heterogeneous rejection. This may explain why some patients with clinical symptoms but negative histological results benefit from immunosuppression. The importance of the uneven distribution of acute rejection exists in: 1, In clinical monitoring of rejection after lung transplantation, choosing susceptible areas may help improve the accuracy of biopsies; 2, Multi-point/multi-lobe drawing can help improve the sensitivity of diagnosis and decrease the potential complications of one-site biopsies, such as bleeding and pneumothorax.

### The significance of interstitial lymphocytes in diagnosing and grading rejection

Although perivascular/peribronchial mononuclear cells infiltration leads to explicit diagnosis of graft rejection, a percentage of clinical cases cannot be diagnosed properly due to failure in obtaining sufficient parenchymal structures from biopsy. Our results demonstrated that quantitative analysis of interstitial T cell infiltration helped evaluate the intensity of acute rejection in transplanted lungs. Tavora and colleagues found in patients undergoing allograft rejection, CD3, CD4 and CD8 T lymphocytes in lung interstitia increased significantly [6]. In this study, interstitial CD3, CD4 and CD8 T cells in the transplanted lungs positively correlated with rejection grading as quantitated with T cell IHC. This suggests that numbering of interstitial T lymphocytes has potential value in monitoring lung transplant rejection. Future studies on utilizing interstitial T cell quantitation to diagnose and grade lung transplant rejection are warranted.

### The auxiliary role of immunohistochemistry in diagnosis of rejection

Fiberbronchoscopic biopsy is presently the ‘gold standard’ for diagnosing and grading lung allograft rejection. There are obvious differences in assessing lung allograft rejection among different medical centers, even different pathologists within the same center [13,14]. H&E staining has certain limitations not only in the diagnosis of rejection but also in the differential diagnosis of rejection from other diseases. The sensitivity and specificity of diagnosis is expected to improve with additional information from special staining techniques such as IHC. This current study showed immunohistochemically stained interstitial T lymphocyte infiltration was easier to identify comparing with sections stained with H&E and thus could help achieve this goal.

Our results were consistent with the study of Tavora and colleagues. T lymphocytes positively stained stood out in sharp contrast against the surrounding background. Diagnosis of lung transplant rejection, which is often overlooked, misgraded, misdiagnosed with conventional H&E examinations, could be improved in sensitivity and specificity [15]. Inconsistency in rejection grading between H&E and IHC mainly existed between grade A1 and A2. This may be related with the following factors: 1, Lesions of grades A1 and A2 are composed of only a small number of mononuclear infiltrates that may be overlooked; 2, As recommended by the International Society of Heart and Lung Transplantation, only cellular infiltrates with circular distribution are valuable in diagnosis. Therefore, there could be, to certain extent, subjectivity in using this diagnostic criteria by different pathologists or by the same pathologist at different times. 3, A few nonspecific aggregated cells interfere with diagnosing processes. This phenomenon demonstrates that on the one hand there are a number of subjective factors in the diagnosis of lung transplant rejection, and on the other hand, it is necessary to use specific staining method to improve the sensitivity and specificity of rejection diagnosis. T lymphocytes quantifications by IHC has some role in helping avoid the interobserver variability in diagnosing and grading lung transplant rejection.

The pathological changes after lung transplantation are complex. Pulmonary complications such as post-transplant lymphoproliferative disorder in the lung are also seen after other solid organ transplantation like kidney transplantion [16-18]. The morphological changes in the lung are diverse; therefore the accurate diagnosis for lung histopathological changes after organ transplantation is very difficult. IHC can provide additional information to aid in diagnosis.

## Conclusions

With orthotopic left lung transplantation model in rats, we found typical rejection in lung allografts. Moreover, rejection in one-third cases heterogeneously distributed in lung allografts, with lesions in the apex and center being more aggravated than those in the base and periphery of lung allografts, respectively. IHC improves the sensitivity and specificity of rejection diagnosis and grading and interstitial T lymphocyte quantitation has potential value in the diagnosing and grading lung allograft rejection.

## Competing interest

The authors declare that they have no competing interest.

## Authors’ contributions

LC and HZG: designed and performed the study, collected data, drafted the paper. XWQ and QL: performed the study, collected data. JN: performed the study, collected data. JSL and JJW: edit the paper. KJ: sponsor, responsible of overall project design, edit the paper. All authors read and approved the final manuscript.

## Authors’ information

Lin Cheng and Haizhou Guo: they should be regarded as co-first authors.
